# Sector-by-sector analysis of dependence dynamics between global large-cap companies and infectious diseases: A time-varying copula approach in EBOV and COVID-19 episodes

**DOI:** 10.1371/journal.pone.0259282

**Published:** 2021-11-03

**Authors:** Mahdi Ghaemi Asl, Hamid Reza Tavakkoli, Muhammad Mahdi Rashidi

**Affiliations:** 1 Faculty of Economics, Kharazmi University, Tehran, Iran; 2 Faculty of Economics, Imam Sadiq University, Tehran, Iran; Beihang University, CHINA

## Abstract

Infectious diseases and widespread outbreaks influence different sectors of the economy, including the stock market. In this article, we investigate the effect of EBOV and COVID-19 outbreaks on stock market indices. We employ time-varying and constant bivariate copula methods to measure the dependence structure between the infectious disease equity market volatility index (IEMV) and the stock market indices of several sectors. The results show that the financial and communication services sectors have the highest and the lowest negative dependency on IEMV during the Ebola virus (EBOV) pandemic, respectively. However, the health care and energy sectors have the highest and lowest negative dependency on IEMV during the COVID-19 outbreak, respectively. Therefore, the results confirm the heterogeneous time-varying dependency between infectious diseases and the stock market indices. The finding of our study contributes to the ongoing literature on the impact of disease outbreaks, especially the novel coronavirus outbreak on global large-cap companies in the stock market.

## 1. Introduction

Infectious disease outbreaks have a significant impact on economic activity. The most recent example is the COVID-19 outbreaks that cause the US economy to shrink by 2.9% at a mild perspective [1]. Since the emergence of COVID-19 in late December, it has infected more than ten million people and killed more than five hundred thousand people worldwide. It forces many people to work from home and the governments to lay restrictions on transportation and travel. The crisis also leads to the economic shutdown and unemployment of millions of people and affected different sectors.

Before COVID-19, two other coronaviruses—SARS-CoV and MERS CoV—also generated worldwide concern due to their global reach and the number of deaths they caused. A devastating EBOV virus (EBOV) outbreak has recently swept through Western Africa. EBOV is a filovirus that causes severe hemorrhagic fever in humans, with up to a 90% case fatality rate if untreated. Outbreaks of EBOV are sporadic, unpredictable, and localized to sub-Saharan Africa [2].

The pandemics affect not only the sectors of the economy but also the economic policies [3]. Several studies investigate the impact of a disease outbreak on the economy separately, which will be presented in the literature review. However, only a few studies like Wilson, Campos [4] and Hassan, Hollander [5] investigate different outbreaks’ economic impacts.

This paper employs the copula method to investigate the dependence structure between stock market indices during the COVID-19 and EBOV outbreaks. For this purpose, we first use the time-varying copula method to extract time-varying and constant dependence structure to all pandemic time. Then, we extract the dependence structure at any time of each pandemic separately. The rest of the paper constructs as follows section 2 present some literature investigating pandemic diseases and the stock market. Section 3 shows the copula-based method and data, and section 4 shows the empirical result, and section 5 outlay the conclusion.

## 2. Literature review

Many studies investigate the effect of the infectious disease outbreak on the different sectors of the economy, especially the stock market. There is plenty of research indicating that pandemics have negatively affected the economy. However, some industries have been affected positively during the pandemic, like high-tech industries. In the following studies that examined the impact of the SARS outbreak, EBOV outbreak, and COVID-19 outbreak on industries and different sectors in the stock markets will be presented.

Chen, Chen [6] investigated the effect of the SARS outbreak on the Taiwan stock market by employing the GARCH and event study approach. The empirical results indicate that SARS affected the tourism industries the biotech industries positively and negatively respectively during the crisis. In addition, Chen, Jang [7] investigate the performance of the hotel industry in the Taiwan stock market during the SARS pandemic by employing the generalized autoregressive conditional heteroskedasticity (GARCH) family models, particularly the exponential GARCH (EGARCH) and the threshold GARCH (TGARCH) methods. The study’s findings confirm the negative impact of the outbreak on the hotel industry. Ichev and Marinč [8] investigated the impact of the EBOV outbreak on investors’ decisions by employing the event study approach and regression models. The results reveal that investors’ decision-making is affected by EBOV.

Recently huge number of studies has investigated the effects of the COVID-19 outbreak on the stock market. For instance Al-Awadhi, Alsaifi [9] investigated the impact of death and confirmed cases of COVID-19 on china’s stock market by employing a panel regression model. The result confirms the negative effect of COVID-19 on all industries in china’s stock market. Onali [10] uses VAR, GARCH, and Markov-Switching with simple regression models to investigate the effects of COVID-19 on the US stock market. The result of the three models confirms the negative impact of the COVID-19 outbreak on Dow Jones and S&P500 returns. The outbreak also positively affects the Dow Jones and S&P500 volatilities; the results also reveal that the COVID-19 outbreak influences these indices in Europe. Yilmazkuday [11] employed the SVAR model and showed that the growth of the COVID-19 outbreak in the US has a negative effect on the S&P 500 Index. Liu, Manzoor [12] employed an event study approach to capture the effect of the COVID-19 on 21 countries’ stock markets, and they come up with the same results. Sharif, Aloui [13] used the wavelet-based approach to analyze the effect of the COVID-19 outbreak and recent oil price volatility on the stock market, geopolitical risk, and economic policy uncertainty in the US. The results reveal that in comparison to oil price volatilities, the COVID-19 outbreak has affected economic uncertainty and geopolitical risk more substantially, and it is projected that the outbreak will have a long-term negative impact on them. However, the recent volatilities in oil prices significantly affect the stock market compared to the COVID-19 outbreak.

He, Liu [14] investigated the direct and spillovers effects of COVID-19 on stock markets in several countries, including the United States, France, Germany, South Korea, and China, and some other countries, by applying conventional t-tests and nonparametric Mann–Whitney tests to daily data of stock markets return. The study’s finding indicates that COVID-19 influences stock markets negatively in short term. The results confirm bidirectional spillover effects between European, American, and Asian stock markets due to impact of the coronavirus outbreak.

Goodell and Huynh [15] investigated the impact of the financial behavior of some legislators who traded stocks from January to February 2020 during the COVID-19 pandemic on financial markets to analyze whether their trades were ahead of the market or not. To this end, they utilized event study methodology to evaluate the response of US industries to sudden COVID-19 announcements. The findings of the study yield two criteria that can determine whether legislators trading were ahead of the market or not. First is trading before February 26, and second trading 15 industries equity with high positive (pharmaceutical and medical products) and negative returns (restaurants, hotels, and motels). These criteria are satisfied by most of the legislators’ trades.

Some research focuses on the impact of coronavirus outbreaks on asset prices like cryptocurrencies and gold, and their safe have properties. For instance, Conlon, Corbet [16] evaluated the safe-haven characteristics of some cryptocurrencies, including Bitcoin, Ethereum, and Tether, during the COVID-19 pandemic by focusing on Value at Risk (VaR) and the corresponding conditional value at risk (CVAR). The empirical results indicate that Bitcoin and Ethereum don’t act as a safe haven for most international equity markets. In contrast, results confirm the safe-haven properties of Tether as its value is pegged to the dollar. Besides, Conlon and McGee [17] analyzed the safe-haven characteristics of Bitcoin during the Covid-19 outbreak by employing the four-moment modified VaR for measuring downside risk. The findings of the study show that bitcoin price decreases during the outbreak. It indicates that bitcoin cannot provide hedging during financial downturns.

In contrast, Goodell and Goutte [18] come up with different results. They investigated the co-movement of bitcoin price and COVID-19 world deaths by applying a wavelet coherence approach to daily data from December 31, 2019, to April 29, 2020. The empirical results indicate that bitcoin prices increased as the crisis developed, especially before April 5, so bitcoin can be considered a safe haven.

The dynamics among the stock indices and cryptocurrencies during the COVID-19 pandemic is also investigated for instance Goodell and Goutte [19] evaluated the effect of COVID-19 on paired co-movement of fourteen equity indices, the volatility index (VIX), and six cryptocurrencies, including bitcoin futures and Tether by employing several econometric methods like principal copula component, neural network analyses, and wavelet coherence. The empirical results indicate that the co-movement between cryptocurrencies and equity indices increases as the crisis develops, and the co-movements are positively correlated except for bitcoin’s future and Tether. It is also shown that equity indices and cryptocurrencies instead of bitcoin’s future and tether prices decrease as the volatility index increases and the outbreak progresses.

Sun, Wu [20] examined the effect of COVID-19 and investor sentiments on the different industries in Chinese stock market by employing an event study approach. Their empirical results indicated that the pandemic affects the stock market negatively generally. In addition, the results reveal that investor sentiments and stock returns are highly correlated during this crisis period. However, some industries, including pharmacy, digitalization, and agriculture, react positively to the pandemic. Xu [21] analyze the interaction between the US and Canada stock return and pandemic uncertainty and changes in the COVID-19 cases by employing the bivariate structural GARCH-in-Mean VAR method. The results reveal that increase in the COVID-19 cases influences the stock market negatively on the whole. In addition, uncertainty negatively impact the US and Canadian stock markets; however, the US stock market is affected to a lesser extent.

Okorie and Lin [22] examined the existence of the COVID-19 pandemic’s fractal contagion effect on the stock markets of 32 countries by employing the Detrended Cross-Correlation Analysis and Detrended Moving Cross-Correlation Analysis methods. The study’s findings indicated that pandemic has a fractal contagion effect on the stock markets of these countries; however, the fractal contagion effect declines gradually in the medium and long terms.

Chang, Feng [23] considered the impact of the reaction of government to the COVID-19 pandemic on the returns of stock markets of 20 countries. The study’s finding reveals that stock market returns are significantly influenced by the government reactions to pandemic. Rahman, Amin [24] investigated the impact of the COVID-19 pandemic on the Australian stock market and the effectiveness of the Government stimulus package in helping the stock market by employing the regression method during COVID-19 crisis. The results indicated that pandemic announcements negatively influenced the stock market, while one of the stimulus packages announcements positively affected the stock market. Their findings also showed that the value portfolios are affected more adversely during the crisis.

Anh and Gan [25] investigate the effect of COVID-19 on Vietnam stock returns using panel-data regression models, and the results indicated that the daily number of COVID-19 cases affect stock returns adversely.

Contessi and De Pace [26] studied the impact of the COVID-19 pandemic on the stock market in 18 countries by employing regression methods, and their results indicated that pandemic caused explosive behavior and affected the stock markets adversely. In addition, the results showed signs of transmission of instability to other stock markets from the Chinese stock market.

Mazur, Dang [27] examined the performance of different industries in the US stock market during the COVID-19 pandemic and, their results indicated that some stocks including, natural gas, food, healthcare, and, software experienced high positive returns. In contrast, other sectors like petroleum, real estate, entertainment, and hospitality crashed sharply. Aloui, Goutte [28] evaluate the impacts of the COVID-19 outbreak on crude oil and natural gas S&P GS Indices by employing the TVP-SVAR with a stochastic volatility model. The study’s finding reveals that the response of energy commodities S&P GS Indices changes over time, depending on financial and fundamental, and behavioral factors. These factors include investors’ expectations, the structural imbalance between supply and demand, and the negative effect of the outbreak on the commodity futures market. Yan, Stuart [29] assessed the impact of coronavirus outbreaks on gold and three industries, including travel, technology, and entertainment, by analyzing the past outbreaks. The results generally indicate that markets respond negatively to outbreaks in the short run, but they will recover in the long run. They suggest that investors can profit by short-selling the industries’ equities as their prices decrease immediately in the short term. They also indicate that buying gold EFTs is a good strategy as gold acts as a safe haven during the crisis.

The result of studies indicated that the disease and pandemics like the COVID-19 pandemic influenced industries and different sectors in the stock markets throughout the world adversely in general. However, there were some exceptions, and as mentioned by Mazur, Dang [27], Sun, Wu [20], and Chen, Chen [6], stock indices of some sectors were affected positively by the pandemic crisis. These stock indices were related to food, healthcare, and information technology industries [30].

## 3. Methodology

The dynamic dependency between IEMV and stock indices is capture by employing a time-varying bivariate copula after constructing the marginal distribution of data. The bivariate copula approach is applied to IEMV and stock market index data that are separated into four periods.

To extract standardized residuals of data, Student’s t ARMA (m, n)-GARCH (1,1) is employed to remove some features that exist in financial time series data, such as volatility clustering. To this end, the GJRGARCH(1,1) model based on the Student’s t introduced by Glosten, Jagannathan [31] is used. The model is defined as follows:

$$\begin{array}{ll} y_{t} & =c+\sigma_{t}z_{t}\\ \sigma_{t}^{2} & =\varsigma_{0}+\varsigma_{1}\varepsilon_{t-1}^{2}+\varsigma_{2}\varepsilon_{t-1}^{2}d_{t-1}+\varsigma_{3}\sigma_{t-1}^{2} \end{array}$$ (1)

Where ε_t_ is residuals of the model with variance σ_t_^2^ and Student’s t innovation distribution, and z_t_ is a random variable with mean 0 and variance 1. The term d_t-1_ is a dummy variable that equals one when ε_t-1_<0 and zero when ε_t-1_>0. ς_2_ implies asymmetric effect when ς_2_≠0 and leverage effect when ς_2_ >0.

The copula is a distribution function that constructs a multivariate joint distribution function. Each copula family has specific marginal distribution and dependence structure. The copula approach is widely used in financial modeling [34, 35] and dependence [32] measuring. Suppose X_t_, Y_t_ is random variables with standard uniform marginal distributions U = F_1_(X_t_), V = F_2_(Y_t_), based on Sklar [33], the joint distribution function of X and Y can be constructed as follow:

$$F(X,Y)=C(F_{1}(X_{t}),F_{2}(Y_{t})),$$ (2)

Where F (X, Y) is the bivariate joint distribution function of X, Y, and C is the copula function ranging from zero to one ([0,1]^2^ interval). The bivariate copula method is a way to measure the dependence structure between two related variables. For this purpose, two popular copula families are applied in financial modeling frequently including Archimedean and Elliptical copula families. In this article, we use variety range of copula functions such as Gaussian, Student’s t, Clayton, Gumbel, Frank, Joe, Clayton-Gumbel (BB1) [34], Joe-Gumbel (BB6), Joe-Clayton (BB7), Joe-Frank (BB8) [35], Tawn [36], rotated copula and survival copula to capture various dependence structures.

Different kinds of dependency coefficients are used in the related literature, such as linear correlation, often recommended for measuring dependencies in econometrics. However, linear correlation is not recommended because of some problems, such as its invariancy under strictly increasing transformations and its dependency on the marginal distribution function. However, rank correlation measures can overcome those problems. This article uses Kendall’s Tau to measure the dependency between variables. Also, Blomqvist’s beta [37] is employed to check the robustness of the results. Additionally, financial data usually show different behavior under the tail. The coefficient of the lower and upper tail dependence can be written as follow:

$$\begin{array}{ll} \xi_{l} & =\xi_{l}(x_{1},x_{2})=\underset{q\to 0}{\text{lim}}\text{P}(x_{2}\leq F_{2}\overset{\leftarrow }{}(q)\left|x_{1}\right.\leq F_{1}\overset{\leftarrow }{}(q)),\\ \xi_{u} & =\xi_{u}(x_{1},x_{2})=\underset{q\to 1}{\text{lim}}\text{P}(x_{2}>F_{2}\overset{\leftarrow }{}(q)\left|x_{1}\right.>F_{1}\overset{\leftarrow }{}(q)), \end{array}$$ (3)

If the calculated ξ_l_ is between zero to one (not equal to zero, ((0,1] interval)) data, have lower tail dependence and similarly, if the obtained ξ_u_ is between zero to one (not equal to zero, ((0,1] interval)) data have upper tail dependence [38].

To capture dynamic dependency between IEMV and stock indices, we apply normal and rotated Gumbel time-varying copula to the whole sample observation. In the estimation of the time-varying normal copula, we consider two steps; first, a copula is estimated with constant parameters, and then it is estimated with time-varying parameters following blow [39]:

$$\theta_{t}=\Gamma (x)\left(\delta_{\theta }+\gamma_{\theta }.\theta_{t-1}+\kappa .\frac{1}{10}\sum_{i=1}^{10}F_{1}{}^{-1}(u_{t-i}).F_{2}{}^{-1}(\nu_{t-i})\right)$$

Moreover, for estimating rotated Gumbel time-varying copula first, we estimate and constant rotated Gumbel copula, and then to capture the time-varying tail dependence coefficient, we compute the following parameters:

$$\theta^{l}{}_{t}=\tilde{\Gamma }(x)\left(\delta^{l}{}_{\theta }+\gamma^{l}{}_{\theta }.\theta^{l}{}_{t-1}+\kappa^{l}.\frac{1}{10}\sum_{i=1}^{10}\left|\left.u_{t-i}-\nu_{t-i}\right|\right.\right)$$

$$\theta^{u}{}_{t}=\tilde{\Gamma }(x)\left(\delta^{u}{}_{\theta }+\gamma^{u}{}_{\theta }.\theta^{u}{}_{t-1}+\kappa^{u}.\frac{1}{10}\sum_{i=1}^{10}\left|\left.u_{t-i}-\nu_{t-i}\right|\right.\right)$$

Where θ_t_ is the time-varying copula parameter. If $\Gamma \left(\text{x}\right)=\frac{1-{\text{e}}^{\text{x}}}{1+{\text{e}}^{\text{x}}}$, and Γ^~^(x) = (1+e^−x^)^-1^, θ_t_ should be in [-1,1] interval. We compare the estimations based on different functions that have been already mentioned and choose a function that yields coefficients with the highest log-likelihood.

There are three methods in estimating copula parameters, including parametric, semi-parametric, and nonparametric. In this article, we use a semi-parametric method to estimate copula parameters. This method is also known as the Canonical Maximum Likelihood (CML) method. Marginal distribution is estimated based on the non-parametrically method. The univariate copula function is estimated by the empirical distribution function that is indicated in the following equation:

$$\begin{array}{l} {\tilde{F}}_{1}(X)=\frac{1}{N+1}\sum_{i=1}^{n}1(X_{ij}\leq x),x\in R.\\ {\tilde{F}}_{2}(Y)=\frac{1}{N+1}\sum_{i=1}^{n}1(Y_{ij}\leq y),y\in R. \end{array}$$ (4)

We apply the empirical distribution functions to the copula function and estimate copula parameters parametrically based on the maximum likelihood method [40]. The following equation shows the maximum likelihood function:

$$\tilde{\Lambda }=\text{arg}\;\underset{\tilde{\Lambda }}{\text{max}}\sum_{t=1}^{T}\text{log}\;c({\tilde{F}}_{1}(X_{t}),{\tilde{F}}_{2}(Y_{t});\Lambda ),$$ (5)

Where Λ^~^ is the vector of copula parameters.

So, first, the residuals of the ARMA-GJR-GARCH model for each variable are extracted, then the empirical distribution function is constructed, and finally, the copula parameters are estimated. The results of dependence structure estimation based on different copula functions (families) are considered, and the function that yields the coefficients with the highest log-likelihood is chosen. Additionally, we use the simulation study to investigate how well the estimations copula functions fit reality.

## 4. Data and results

Assessing the economic impact of the COVID-19 pandemic is essential for investors, regulators, and academics, but it is challenging as the crisis has not been fully unfolded yet, and the future perspectives are not clear. Baker, Bloom [41] identified three indicators including stock market volatility, newspaper-based economic uncertainty, and subjective uncertainty in business expectation surveys that provide real-time forward-looking uncertainty measures. They use these indicators to document and quantify the severe spike in economic uncertainty in the past several weeks during the coronavirus outbreak. However, in this study, we employ the infectious disease equity market volatility index (IEMV) to measure dynamic dependency between the uncertainty of pandemics and stock market indices in the last decade.

The data in our study are daily return of eleven sectoral stock indices of global large-cap companies and IEMV spanning from 05/03/2010 to 04/05/2021. The logarithmic form of the IEMV and stock market index return is used in the time-varying bivariate copula model to capture the dependence structure between IEMV and sectoral indices. For estimating constant bivariate copula, data are separated into four periods: pre-EBOV, during EBOV pandemic, pre-COVID-19, and during COVID-19 pandemic. The corresponding date for each period is depicted in Table 1.

**Table 1:** Four periods of data.

period	date
pre-EBOV	05/03/2010 to 03/23/2014
EBOV	03/24/2014 to 10/31/2016
pre-COVID-19	11/01/2016 to 01/20/2020
COVID-19	01/21/2020 to 04/05/2021

The IEMV data are obtained from the Federal Reserve Bank of St. Louis (FRED) website (https://fred.stlouisfed.org/series/infectdisemvtrackd.). The data of sectoral stock market indices are extracted from https://us.spindices.com/. Data consists of stock market indices of eleven sectors, including materials, industrials, consumer discretionary, utilities, communication services, health care, consumer staples, information technology, financials, carbon-efficient, and energy. These sectors are members of the S&P Global 1200 classified within the GICS, including large-cap stocks from major markets worldwide. The S&P Global 1200 provides efficient exposure to the global equity market. It is constructed as a composite of 7 headline indices, many of which are accepted leaders in their regions. These include the S&P 500^®^ (US), S&P Europe 350, S&P TOPIX 150 (Japan), S&P/TSX 60 (Canada), S&P/ASX All Australian 50, S&P Asia 50 and S&P Latin America 40. The database could be found at: https://ndownloader.figshare.com/files/27846798. The descriptive statistics of data in each period are presented in Table 2. The IEMV has the highest kurtosis value (during the COVID-19 pandemic), followed by financial (during the EBOV outbreak). The Jarque-Bera statistics for each variable are rejected in all periods, confirming that data are not normally distributed. Several unit root tests, including Augmented Dicky-Fuller (ADF), Phillips-Perron (PP), and Kwiatkowski–Phillips–Schmidt–Shin (KPSS), are employed to check the stationarity of data. The null hypothesis of non-stationarity is rejected for all returns in each period, which implies that all series are stationary.

**Table 2:** Descriptive statistics of indices returns.

Variables	Mean	Max.	Min.	Std. Dev.	Skewness	Kurtosis	Jarque Bera	ADF	PP	KPSS
**Pre-EBOV**										
Materials	0.0008	5.6899	-6.8627	1.2861	-0.2170	5.9898	384.874***	-26.510***	-26.113***	0.050
Industrials	0.0341	4.8544	-5.6445	1.0988	-0.3610	6.3648	499.385***	-27.819***	-27.602***	0.105
Consumer Discretionary	0.0509	4.4023	-5.6670	1.0124	-0.5030	6.4387	541.293***	-19.524***	-27.265***	0.097
Utilities	0.0052	3.5381	-4.4557	0.8719	-0.2897	5.2788	233.117***	-30.123***	-30.290***	0.101
Communication Services	0.0247	4.1031	-3.7215	0.8402	-0.1980	5.0669	186.751***	-29.989***	-30.116***	0.048
Health Care	0.0585	3.4677	-4.3695	0.8376	-0.5153	6.1699	468.485***	-31.560***	-31.614***	0.161
Consumer Staples	0.0381	3.1990	-3.3674	0.7308	-0.3185	5.3374	247.487***	-31.034***	-31.146***	0.030
Information Technology	0.0357	4.0359	-5.3203	1.0200	-0.2808	5.7758	338.191***	-28.780***	-28.658***	0.085
Financials	0.0181	6.9536	-6.5830	1.2795	-0.1672	6.8308	623.516***	-28.878***	-28.794***	0.19
Carbon Efficients	0.0307	5.0145	-5.2743	0.9925	-0.3518	6.7036	599.266***	-28.330***	-28.224***	0.084
Energy	0.0171	4.8507	-6.7925	1.2353	-0.4127	6.2251	467.319***	-29.437***	-29.364***	0.037
IEMV	2.3209	242.7748	-230.025	78.1820	0.1502	3.5374	2.3686	-5.579***	-12.729***	0.063
**EBOV**										
Materials	-0.0179	3.3188	-5.6423	1.0052	-0.3851	5.1820	151.2515***	-20.880***	-20.642***	0.145
Industrials	0.0059	2.6743	-5.4341	0.7778	-0.7025	7.1804	549.4637***	-21.613***	-21.259***	0.040
Consumer Discretionary	0.0119	2.6720	-5.4697	0.7962	-0.8947	7.3749	631.171***	-21.238***	-20.811***	0.055
Utilities	0.0017	2.9241	-3.9990	0.7870	-0.5933	5.1901	175.2836***	-25.135***	-25.136***	0.036
Communication Services	-0.0056	2.8743	-4.4561	0.7425	-0.3338	6.3438	328.458***	-23.222***	-23.128***	0.057
Health Care	0.0098	2.6118	-3.5464	0.8394	-0.3967	4.4484	77.04007***	-23.786***	-23.758***	0.241
Consumer Staples	0.0189	2.2042	-3.3561	0.6685	-0.4087	5.3180	170.658***	-24.116***	-24.049***	0.050
Information Technology	0.0398	3.9858	-4.4156	0.8982	-0.4827	5.8939	262.920***	-22.739***	-22.549***	0.049
Financials	-0.0087	2.7832	-7.8568	0.9345	-1.2647	11.7195	2328.57***	-22.192***	-21.915***	0.059
Carbon Efficients	0.0038	2.5731	-5.0686	0.7670	-0.7441	7.2765	579.209***	-21.899***	-21.592***	0.048
Energy	-0.0405	4.9182	-5.5986	1.3429	-0.0947	4.6327	76.3200***	-22.988***	-22.893***	0.114
IEMV	-0.0646	262.340	-304.054	98.2358	-0.2092	3.6586	5.52980*	-10.038***	-24.804***	0.031
**Pre-COVID-19**										
Materials	0.0303	3.1467	-2.7524	0.7886	-0.1851	3.8947	32.6543***	-24.050***	-24.056***	0.151
Industrials	0.0403	2.5474	-3.2754	0.6866	-0.6057	5.3998	251.72***	-23.883***	-23.866***	0.124
Consumer Discretionary	0.0462	3.5579	-3.0030	0.7086	-0.3766	5.6907	271.948***	-25.562***	-25.562***	0.077
Utilities	0.0344	2.1557	-3.1315	0.6227	-0.6190	4.8387	171.146***	-21.730***	-26.225***	0.127
Communication Services	0.0153	3.4474	-3.4268	0.7185	-0.2285	5.4885	222.994***	-25.755***	-25.597***	0.170
Health Care	0.0508	3.0663	-3.7501	0.7022	-0.4351	5.9200	323.387***	-25.046***	-24.840***	0.065
Consumer Staples	0.0208	1.9312	-3.0470	0.5597	-0.6970	5.4819	282.255***	-25.147***	-24.977***	0.089
Information Technology	0.0855	4.5175	-4.5663	0.9771	-0.6619	6.1546	407.685***	-27.502***	-27.497***	0.107
Financials	0.0347	2.9348	-3.2684	0.7395	-0.3785	5.1318	178.259***	-24.408***	-24.549***	0.237
Carbon Efficients	0.0439	2.8717	-3.1167	0.6140	-0.6596	6.5415	497.500***	-25.087***	-25.036***	0.104
Energy	-0.0024	4.1184	-3.5749	0.9685	-0.2514	4.3798	75.1296***	-26.209***	-26.209***	0.069
IEMV	2.6403	173.9574	-184.845	71.3014	-0.0818	2.7269	0.59110	-10.282***	-10.308***	0.085
**COVID-19**										
Materials	-0.2446	9.7589	-10.8049	2.8926	-0.5082	6.2160	37.91862***	-9.093***	-9.149***	0.202
Industrials	-0.3656	9.6256	-10.4744	2.9397	-0.3058	5.8270	27.88647***	-8.784***	-8.866***	0.153
Consumer Discretionary	-0.1716	7.9781	-9.7837	2.6932	-0.7622	6.4856	48.24451***	-4.588***	-9.256***	0.194
Utilities	-0.2346	9.1063	-11.8395	3.2426	-0.2445	5.4067	20.10497***	-5.007***	-9.780***	0.076
Communication Services	-0.1287	5.8979	-9.0262	2.5322	-0.6764	5.6295	29.14791***	-13.017***	-12.194***	0.258
Health Care	-0.0587	6.3135	-8.1023	2.4790	-0.2696	4.5617	9.09890**	-5.175***	-10.860***	0.213
Consumer Staples	-0.1460	5.5053	-8.9211	2.1549	-0.5375	6.1948	37.87409***	-10.338***	-10.310***	0.148
Information Technology	-0.0717	9.5976	-12.8240	3.4585	-0.3645	5.5925	24.1746***	-13.393***	-12.731***	0.198
Financials	-0.4611	10.6715	-11.6125	3.4713	-0.5142	5.7936	29.53976***	-10.779***	-10.581***	0.133
Carbon Efficients	-0.2152	8.5413	-10.4486	2.9410	-0.6237	5.8997	33.21426***	-5.359***	-11.149***	0.189
Energy	-0.5748	15.5220	-21.3370	4.9631	-1.0897	7.9409	97.20717***	-9.451***	-9.531***	0.190
IEMV	2.8433	351.4739	-301.489	73.3491	0.6061	12.3571	270.785***	-13.882***	-15.434***	0.232

*, ** and *** indicate significance at the 10%, 5% and 1% level, respectively.

Source: author’s calculation.

Kendall plots (K-plot) are used to visualize the dependency of sectoral indices on IEMV. The results are depicted in Fig 1. It is evident that the decadency changes over time during EBOV and COVID-19 periods, and negative dependency prevail, but during pre- EBOV and pre- COVID-19 positive dependencies are dominant.

**Fig 1:** Kendall plot (K-plot) results for bivariate copula. This shows the dependency of sectoral indices on IEMV (https://ndownloader.figshare.com/files/29099883).

To obtain standardized residuals from time series, ARMA (1,1)-GJR-GARCH (1,1) based on Student’s t distribution is applied to time series returns. To check the serial correlation and ARCH effects in residuals, the Ljung-Box and ARCH-LM tests are carried out. The results confirm that there is no serial correlation and ARCH effect in residuals.

For measuring the constant dependence coefficient between IEMV and other sectoral index data, we apply the Normal and Rotated Gumbel time-varying copula method to whole sample data ranging from 2010 to 2021. Table 3 represents the dependency coefficients obtained from the normal and Rotated Gumbel time-varying copula models and their corresponding log-likelihood and Akaike information criterion [28]. According to log-likelihood and AIC results, the best-fitted copula approach is the Normal time-varying copula, as shown in Fig 2. Based on Normal time-varying copula results shown in Table 3, there is a negative dependency between IEMV and all sectoral stock market indices except for stock indices of communication services and energy sectors. Besides, the health care sector has the highest dependency on IEMV.

**Fig 2:** Time-varying and constant normal copula results. This figure shows the results of the normal time-varying copula, implying there is a negative dependency between IEMV and sectoral stock market indices except for communication services and energy sectors. Besides, the health care sector has the highest dependency on IEMV (https://ndownloader.figshare.com/files/29099883).

**Table 3:** Time-varying copula results.

Sector	Time-varying Normal			Rotated Gumbel		
	Constant ρ	Log-likelihood	AIC	Constant tau	Log-likelihood	AIC
Energy	0.0114566	-1.6487849	0.6424148	1.4972504	-312.109396	0.09275645
Carbon Efficient	-0.002449	-0.2017943	0.8524891	1.48560081	-297.822127	0.76217924
Financials	-0.0082573	-1.19674	0.0479853	1.480562	-294.06535577	0.02587467
Information Technology	-0.0018127	-0.006454	0.6739275	1.48917129	-301.8988812	0.01479562
Consumer Staples	-0.0035907	-0.1347898	0.9149677	1.49115936	-303.234450	0.6458971
Health Care	-0.019961	-1.1118731	0.5746951	1.48870722	-301.8716654	0.4987655
Communication Services	0.00702536	-0.2442827	0.3789417	1.4992391	-314.5757673	0.00587464
Utilities	-0.0175742	-0.9385758	0.1096515	1.48105794	-299.6565285	0.04897274
Consumer Discretionary	-0.006494	-0.3202215	0.4298751	1.47696439	-295.9617135	0.08794789
Industrials	-0.0046432	-0.517580	0.0591764	1.48230050	-300.009660	0.00211758
Materials	-0.0125473	-0.468179	0.4475617	1.473963773	-282.698499	0.30154867

Source: author’s calculation.

Then the bivariate copula parameters are estimated for each of the four observation periods by employing different copula functions. The models with the highest log-likelihood are selected. Tables 4 to 7 represent the results of the selected copula model and the corresponding copula families for every four periods.

**Table 4:** Copula results during the Pre-EBOV period.

Sector	Par1	Par2	Family	Tau	LTD	UPD	LL	IT	AIC
Energy	0.0385	17.4257	*t*	0.0245	0.0006	0.0006	1.8850	0.2016	0.2300
Carbon Efficient	0.0490	18.9611	*t*	0.0312	0.0004	0.0004	2.2369	0.1258	-0.4738
Financials	0.0638	17.0077	*t*	0.0407	0.0009	0.0009	3.5489	0.0527	-3.0978
Information Technology	0.0441	20.7068	*t*	0.0281	0.0002	0.0002	1.9765	0.2029	0.0470
Consumer Staples	1.0552	1.0000	*BB8*	0.0309	0.0000	0.0712	3.2053	0.2595	-2.4106
Health Care	1.0681	0.9816	*BB8*	0.0321	0.0000	0.0000	2.3146	0.2203	-0.6293
Communication Services	0.0345	11.3892	*t*	0.0219	0.0050	0.0050	3.7113	0.2627	-3.4226
Utilities	1.0598	0.9944	*BB8*	0.0312	0.0000	0.0000	2.6504	0.1968	-1.3008
Consumer Discretionary	1.1427	0.0799	*Tawn type 2*	0.0247	0.0000	0.0313	2.4487	0.2087	-0.8974
Industrials	0.0828	0.0000	*Survival Clayton*	0.0398	0.0000	0.0002	3.0222	0.1353	-4.0444
Materials	0.0263	15.6300	*t*	0.0167	0.0010	0.0010	1.8230	0.3989	0.35410

Note: par1, par2 shows estimated copula parameters. Tau is Kendall’s tau coefficient, estimated from the bivariate copula function. LTD, UPD, LL, IT, and AIC indicate the lower tail dependency, the upper tail dependency, the log-likelihood value, the independency test, and Akaike’s information criterion, respectively. Source: author’s calculation.

**Table 5:** Copula results during the EBOV period.

Sector	Par1	Par2	Family	Tau	LTD	UPD	LL	IT	AIC
Energy	-6.9463	0.0057	*Rotated Tawn type 2 90 degrees*	-0.0057	0.0000	0.0000	3.4981	0.7715	-2.9963
Carbon Efficient	-2.3940	0.0110	*Rotated Tawn type 2 90 degrees*	-0.0108	0.0000	0.0000	2.1698	0.2204	-0.3396
Financials	-0.4957	0.0000	*Frank*	-0.0545	0.0000	0.0000	2.3227	0.0322	-2.6454
Information Technology	-1.5661	0.0148	*Rotated Tawn type 2 90 degrees*	-0.0127	0.0000	0.0000	1.1980	0.7973	1.6039
Consumer Staples	-1.5271	0.0256	*Rotated Tawn type 2 90 degrees*	-0.0206	0.0000	0.0000	2.1178	0.3886	-0.2356
Health Care	-2.3577	0.0252	*Rotated Tawn type 2 90 degrees*	-0.0241	0.0000	0.0000	5.4047	0.5072	-6.8094
Communication Services	-4.4002	0.0027	*Rotated Tawn type 2 270 degrees*	-0.0018	0.0000	0.0000	0.6851	0.6756	2.6298
Utilities	-3.2090	0.0111	*Rotated Tawn type 1 270 degrees*	-0.0110	0.0000	0.0000	3.3821	0.1616	-2.7641
Consumer Discretionary	-1.1148	-0.9341	*Rotated BB8 270 degrees*	-0.0414	0.0000	0.0000	1.9117	0.0917	0.1767
Industrials	-0.3426	0.0000	*Frank*	-0.0377	0.0000	0.0000	1.1187	0.1360	-0.2374
Materials	-1.5069	0.0348	*Rotated Tawn type 1 270 degrees*	-0.0267	0.0000	0.0000	2.6730	0.2483	-1.3460

Note: see note of Table 4.

**Table 6:** Copula results during the Pre-COVID-19 period.

Sector	Par1	Par2	Family	Tau	LTD	UPD	LL	IT	AIC
Energy	20.0000	0.0027	*Tawn type 1*	0.0000	0.0000	0.0027	4.4058	0.7753	-4.8117
Carbon Efficient	0.0227	27.6897	*t*	0.0144	0.0000	0.0000	0.6557	0.4898	2.6885
Financials	15.1233	0.0030	*Rotated Tawn type 2 180 degrees*	0.0000	0.0030	0.0000	4.4429	0.5010	-4.8858
Information Technology	13.3279	0.0023	*Rotated Tawn type 2 180 degrees*	0.0000	0.0023	0.0000	2.2011	0.8952	-0.4022
Consumer Staples	7.0548	0.0024	*Rotated Tawn type 1 180 degrees*	0.0024	0.0024	0.0000	1.9978	0.6233	0.0045
Health Care	1.2713	0.0336	*Rotated Tawn type 1 180 degrees*	0.0194	0.0231	0.0000	1.3616	0.3124	1.2768
Communication Services	1.0658	0.1993	*Tawn type 2*	0.0241	0.0000	0.0320	1.2771	0.1921	1.4458
Utilities	20.0000	0.0017	*Rotated Tawn type 2 180 degrees*	0.0000	0.0017	0.0000	0.9245	0.6573	2.1509
Consumer Discretionary	1.0172	0.0000	*Survival Joe*	0.0099	0.0234	0.0000	0.1926	0.8630	1.6148
Industrials	20.0000	0.0013	*Rotated Tawn type 2 180 degrees*	0.0000	0.0013	0.0000	0.2995	0.6032	3.4010
Materials	-1.0264	0.0000	*Rotated Joe 90 degrees*	-0.0150	0.0000	0.0000	0.7124	0.8415	0.5751

Note: see note of Table 4.

**Table 7:** Copula results during the COVID-19 period.

Sector	Par1	Par2	Family	Tau	LTD	UPD	LL	IT	AIC
Energy	-13.2336	0.0579	*Rotated Tawn type 2 90 degrees*	-0.0576	0.0000	0.0000	3.4116	0.3366	-2.8232
Carbon Efficient	-1.6161	0.2090	*Rotated Tawn type 2 90 degrees*	-0.1280	0.0000	0.0000	2.7268	0.1513	-1.4536
Financials	-1.6076	0.2348	*Rotated Tawn type 2 90 degrees*	-0.1390	0.0000	0.0000	2.5645	0.2513	-1.1290
Information Technology	-1.2402	-1.0000	*Rotated BB8 90 degrees*	-0.1204	0.0000	0.0000	2.0399	0.1163	-0.0797
Consumer Staples	-1.6260	0.2345	*Rotated Tawn type 2 90 degrees*	-0.1409	0.0000	0.0000	3.1257	0.0471	-2.2515
Health Care	-1.2892	-1.0000	*Rotated BB8 90 degrees*	-0.1411	0.0000	0.0000	2.9142	0.1561	-1.8284
Communication Services	-4.8156	0.0766	*Rotated Tawn type 2 90 degrees*	-0.0747	0.0000	0.0000	2.8227	0.3855	-1.6453
Utilities	-9.8532	0.0921	*Rotated Tawn type 2 90 degrees*	-0.0911	0.0000	0.0000	5.1386	0.0979	-6.2772
Consumer Discretionary	-2.7222	0.0686	*Rotated Tawn type 2 90 degrees*	-0.0641	0.0000	0.0000	1.4670	0.4486	1.0659
Industrials	-1.6168	0.2334	*Rotated Tawn type 2 90 degrees*	-0.1394	0.0000	0.0000	2.9246	0.2766	-1.8492
Materials	-1.9413	0.1485	*Rotated Tawn type 2 90 degrees*	-0.1143	0.0000	0.0000	2.5677	0.3323	-1.1355

Note: see note of Table 4.

Tables 4–7 are summarized in Fig 3 and Table 8. The results indicate that there is a negative dependency between IEMV and other sectoral stock market indices during EBOV and COVID-19 periods, but the dependency during the coronavirus outbreak is much higher. The results also confirm that there is a positive dependency between IEMV and other sectoral stock indices during Pre-EBOV and Pre-COVID-19 eras except for material, which indicates negative dependency with IEMV during the pre-COVID-19 period. Therefore, as the volatilities related to infectious disease in the stock market spike during pandemics, the sector stock indices plunge, so we face high negative dependency between IEMV and stock indices, especially during the COVID-19 pandemic. This result is supported by Al-Awadhi, Alsaifi [9], Onali [10], Yilmazkuday [11], Liu, Manzoor [12], Sharif, Aloui [13], He, Liu [14], and Yan, Stuart [29] who showed a negative impact of COVID-19 on stock indices.

**Fig 3:** Dependency analysis during episodes. This plot indicates that there is a high negative dependency between IEMV and other sectoral stock market indices during EBOV and COVID-19 periods, but the dependency during the coronavirus outbreak is much higher (https://ndownloader.figshare.com/files/29099883).

**Table 8:** Summary of dependency on IEMV during episodes.

	Maximum Positive Dependency	Minimum Positive Dependency	Highest Negative Dependency	Lowest Negative Dependency
Pre-EBOV	Financials (0.04)	Materials (0.01)	-	-
EBOV	-	-	Financials (-0.05)	Communication Services (-0.001)
Pre-COVID-19	Communication Services (0.024)	Industrials (3.3E-09)	Materials (-0.01)	Materials (-0.01)
COVID-19	-	-	Health Care (-0.14)	Energy (-0.05)

Note: Numbers in parentheses are the dependency coefficients.

However, during the pre-outbreak periods when the IEMV is very low or near zero, the dependency is positive, implying that most stock prices respond positively to very low values of IEMV, especially during the pre-EBOV period. It is also evident that some sectors like industries, utilities, information technology, financials, and energy are not affected by IEMV during pre-COVID-19.

Table 8 shows the sectors with the highest and lowest dependency on IEMV during every four periods. In the pre-EBOV era, financials, industries, and health care had the highest positive dependencies with IEMV. Besides, during the EBOV era, financials, consumer discretionary, and industrials had the highest negative dependencies with IEMV, meaning that IEMV greatly influences these sectors during this period. In contrast, communication services and energy were affected the least. During the pre-COVID-19 era, communication services and health care showed the highest dependency on IEMV. During the COVID-19 outbreak, industrials, health care, consumer staple, and financials have the highest negative dependency on IEMV, implying that these sectors suffer the most from the COVID-19 pandemic. In contrast, energy, consumer discretionary, and communication services indicate a minor dependency on IEMV.

It is noteworthy that communication services are among the least affected sectors during both outbreaks. Since, during pandemics, as more people telework and the government lay restrictions on commuting, the demand for communication services increases, mitigating the negative effects of the outbreak on communication services. The energy sector that was positioned to be the least affected sector during these two outbreaks was more influenced during COVID-19 due to economic shutdowns and restrictions on travel and transportation.

Both industrials and financials sectors are profoundly affected during both outbreaks because of a decrease in investments and manufacturing activities due to economic shutdown and consequent rescission. This result is in line with Al-Awadhi, Alsaifi [9], who found that the COVID-19 outbreak had a negative impact on industries in China.

Scatter plots and Contour plots are employed to better illustrate the relationship between each sectoral index and IEMV. Figs 4 and 5 represent the scatter plot and Contour plot of the bivariate copula for every four periods. The figures confirm the asymmetry and tail dependence in joint distribution at pre-EBOV and pre-COVID-19 periods.

**Fig 4:** Scatter plot of each bivariate copula function for every four periods. The plot confirms the asymmetry and tail dependence in joint distribution at pre-EBOV and pre-COVID-19 periods *(*https://ndownloader.figshare.com/files/29099883).

**Fig 5:** Contour plot of each bivariate copula function for every four periods. The contour plot of the bivariate copula highlights the asymmetry and tail dependence in joint distribution at pre-EBOV and pre-COVID-19 periods *(*https://ndownloader.figshare.com/files/29099883).

We also simulated data from selected copula functions and compared them with the real data to evaluate how well-fitted our estimations are. The results are represented in Fig 6. The red point indicates the observation data, and the blue point shows the simulated data. The results confirm that the generated data through the simulation process from copula functions are very close to observation data except for the pre-COVID-19 period. In the pre-COVID-19 period, some extreme returns are not captured by the simulation process.

**Fig 6:** Simulation of each bivariate copula function for every four periods. The red point indicates the observation data, and the blue point shows the simulated data. The results confirm that the generated data through the simulation process from copula functions are very close to observation data except for the pre-COVID-19 period (https://ndownloader.figshare.com/files/29099883).

## 5. Robustness test

To check the robustness of the results, we try to estimate the bivariate copula parameter using Blomqvist’s beta for EBOV and COVID-19 periods. Then we compare the obtained coefficients with the Tau coefficient of the bivariate copula. The results are presented in Table 9 and Fig 7. The results indicate that Blomqvist’s beta coefficients and Tau coefficients are close to each other, implying the robustness of the results.

**Fig 7:** Compare Kendall’s tau and Blomqvist’s beta coefficient of bivariate copula for EBOV and COVID-19 periods. The results indicate that Blomqvist’s beta coefficients and Tau coefficients are close to each other, implying the robustness of the results (https://ndownloader.figshare.com/files/29099883).

**Table 9:** The result of Kendall’s tau and Blomqvist’s beta coefficients of bivariate copula for EBOV and COVID-19 periods.

	EBOV		COVID-19	
	Tau	Beta	Tau	Beta
Energy	-0.0057	-0.0039	-0.0576	-0.0410
Carbon Efficient	-0.0108	-0.0076	-0.1280	-0.1176
Financials	-0.0545	-0.0618	-0.1390	-0.1292
Information Technology	-0.0127	-0.0097	-0.1204	-0.1128
Consumer Staples	-0.0206	-0.0162	-0.1409	-0.1308
Health Care	-0.0241	-0.0175	-0.1411	-0.1331
Communication Services	-0.0018	-0.0019	-0.0747	-0.0545
Utilities	-0.0110	-0.0077	-0.0911	-0.0659
Consumer Discretionary	-0.0414	-0.0417	-0.0641	-0.0486
Industrials	-0.0377	-0.0428	-0.1394	-0.1294
Materials	-0.0267	-0.0214	-0.1143	-0.0988

## 6. Diversification analysis

After finding the relationship between IEVM and stock indices of different sectors, in this section, we want to explore the implications of their relationships on optimal portfolio weight strategy.

The optimal weight of sector stock indices in a one-dollar portfolio of infectious disease equity market volatility index (IEMV) can be computed using the estimated conditional variance-covariance. The optimal weight of y in a one-dollar portfolio of x can be shown as follows:

$${\text{w}}_{\text{yx},\text{t}}=\frac{{\text{h}}_{\text{xx},\text{t}}-{\text{h}}_{\text{xy},\text{t}}}{{\text{h}}_{\text{yy},\text{t}}-2{\text{h}}_{\text{xy},\text{t}}+{\text{h}}_{\text{xx},\text{t}}}$$

$$w_{yx,t}\left\{\begin{array}{ll} 0 & w_{yx,t}<0\\ w_{yx,t} & 0\leq w_{yx,t}\leq 1\\ 1 & w_{yx,t}>1 \end{array}\right.$$

Where *w*_*yx*,*t*_ indicate the weight of y in a one-dollar portfolio of x and h_xy_ is the conditional covariance between x and y and h_xx_ and h_yy_ are the conditional variance of x and y, respectively. After constructing a portfolio based on the optimal weights, we compare the variance of hedged and unhedged portfolios represented by *Var*_*hedged*_ and *Var*_*unhedged*_ respectively and defined the hedging effectiveness as follows:

$$\text{HE}=\;\frac{{\text{Var}}_{\text{unhedged}}-{\text{Var}}_{\text{hedged}}}{{\text{Var}}_{\text{unhedged}}}\times 100$$

The portfolio weights and hedging effectiveness results are indicated in Tables 10 and 11. Also, the results are depicted graphically in Figs 8 and 9.

**Fig 8:** Dynamic optimal weights strategy results. Time-varying optimal weights of each sectoral indices in the IEMV-sectoral index diversified portfolios (https://ndownloader.figshare.com/files/29099883).

**Fig 9:** Effectiveness of optimal weights strategy. Dynamic effectiveness of diversifying IEMV with each sectoral indices (https://ndownloader.figshare.com/files/29099883).

**Table 10:** Optimal weights of sectoral indices in the IEMV-sectoral index diversified portfolios.

Episode	Materials	Industrials	Consumer Discretionary	Utilities	Communication Services	Health Care	Consumer Staples	Information Technology	Financials	Carbon Efficients	Energy
Pre-EBOV	9.278	10.148	3.952	6.815	2.816	5.803	3.769	0.341	13.051	4.179	16.939
EBOV	8.806	9.800	3.680	6.654	2.693	5.742	3.683	0.157	12.550	3.997	16.923
Pre-COVID	8.679	9.847	3.656	6.591	2.711	5.676	3.652	0.242	12.496	3.968	16.616
COVID	2.486	2.861	1.055	1.906	0.813	1.587	0.986	0.292	3.770	1.101	5.496

**Table 11:** Effectiveness of diversifying IEMV with each sectoral indices.

Episode	Materials	Industrials	Consumer Discretionary	Utilities	Communication Services	Health Care	Consumer Staples	Information Technology	Financials	Carbon Efficients	Energy
Pre-EBOV	0.940	1.976	0.016	0.659	-0.046	0.450	0.161	-0.034	3.223	0.110	3.586
EBOV	0.852	1.872	0.002	0.632	-0.046	0.440	0.154	-0.022	3.055	0.093	3.571
Pre-COVID	0.831	1.892	0.000	0.623	-0.047	0.431	0.151	-0.033	3.049	0.089	3.490
COVID	0.109	0.247	0.001	0.080	0.000	0.054	0.020	-0.008	0.406	0.012	0.565

The computed optimal weight indicates the optimal weights of sectoral stock indices in a portfolio of IEMV, and each stock indices do not change during Pre-EBOV, EBOV, and Pre-COVID periods; however, they plunged during COVID, implying that during the COVID pandemic, the optimal portfolio should consist of more IEMV to minimize the risk. Besides, the diversification cost of a portfolio consisted of IEMV decrease during the COVID-19 crisis. In addition, adding the stock indices of the Information Technology sector and the energy sector are the least and most costly way to build a portfolio of IEMV and each sectoral stock indices during these periods. The results of hedging effectiveness are shown in Table 11. The result indicated that during the COVID-19 period, the hedge effectiveness of most of the hedged portfolios decrease, showing that the optimal weight strategy becomes less effective during the pandemic crisis due to high turmoil in the stock market. While during the Pre-EBOV, EBOV, and Pre-COVID periods hedging effectiveness are constant for optimal portfolios. Finally, stock indices energy, financial, and materials are the most effective assets to diversify the portfolio. While adding stock indices of Consumer Discretionary, Communication Services, Information Technology for diversification purposes is not recommended.

## 7. Conclusion

This paper investigates the dependence structure between eleven sectoral stock market indices and the infectious disease equity market volatility index (IEMV) by applying the copula framework to four sample periods, namely pre-EBOV, during the EBOV pandemic pre-COVID-19, and the COVID-19 pandemic. Before applying the time-varying copula to capture the dynamic structure of the dependence coefficient between IEMV and other stock indices, the marginal distribution of data is constructed by employing the Student’s t ARMA (1,1)-GARCH (1,1) model. Besides, the bivariate copula is also estimated for every four periods. The results confirm tail dependence in data during pre-EBOV and pre-COVID-19 periods and the negative dependence between IEMV and sectoral indices during EBOV and COVID-19 periods. It is also found that there is a positive dependency between IEMV and most of the sectoral indices during the Pre- EBOV and Pre-COVID-19 periods.

Throughout the EBOV period, financials, consumer discretionary, and industrials had the highest negative dependency IEMV. The negative dependency between IEMV and other sectoral indices significantly rise during the COVID-19 period compared to the EBOV period implying that COVID-19 has influenced the stock market more significantly than the EBOV. Industrials, health care, consumer staple, financials had the highest negative dependency on IEMV during this period.

On the other hand, over the EBOA outbreak period, the communication services sector and the energy sector had the least dependency on IEMV, while during the COVID-19 outbreak, energy, consumer discretionary, and communication services have had the lowest correlation with IEVM.

A comprehensive comparison of the dependence between IEMV and stock indices of different sectors during EBOV outbreaks and the COVID-19 pandemic can yield interesting implications. First, during the COVID-19 period, there is a much higher dependency between IEMV and sectoral stock indices compared to the EBOLA period. This is due to the fact that COVID-19 has affeered almost every country and every sector in the world while the EBOLA outbreak was restricted to some regions. So, it is reasonable to see that stock indices have higher negative dependency during the period. Second, Financials and industrials were both among the sectors that have negative dependency on IEMV throughout EBOV and COVID-19 periods. However, the dependency between indices surged during the COVID-19 era. This can be due to the negative effect of the COVID-19 pandemic on investments and manufacturing sectors, as many countries face economic shutdowns and economies plunge into recession. Third, on the other hand, Communication services were among the sectors that have the least dependency on the IEMV during these two outbreaks, implying that these companies’ performance is relativity less connected to outbreaks due to special features of services they offer.

Finally, the diversification implications of the dependence between IEMV and sectoral stock indices are investigated by computing portfolio weights and hedging effectiveness. The computed optimal weight indicates the optimal weights of sectoral stock indices in a portfolio of IEMV, and each stock index is much lower during COVID than pre-EBOV, EBOV, and Pre-COVID periods, implying a decrease in diversification costs. The results of hedging effectiveness indicated that the hedge effectiveness of most of the hedged portfolios decrease during the COVID-19 period implying that the optimal weight strategy becomes less effective during the COVID-19 pandemic. This result can be related to the disturbance in the stock market caused by the COVID-19 pandemic. The results can be beneficial for academics, investors, and policymakers. The study also contributes to the literature on the economic effects of disease outbreaks, specifically the COVID-19. On the top of the list of the suggestions for future works, we could consider volatility clustering, which simply can be described as irregular changing between high volatility and low volatility trends. It is a common feature of financial data, so future studies can investigate the diversification and hedging strategies allowing for volatility clustering that can be computed using different approaches that have been proposed by following [42–46].

## Abbreviations

ADF: Augmented Dicky-Fuller
ARCH-LM: Autoregressive Conditional Heteroscedasticity-Lagrange Multiplier
ARMA: Autoregressive–Moving-Average
CVAR: Conditional Value at Risk
EBOV: EBOV virus
EGARCH: Exponential GARCH
FRED: Federal Reserve Bank of St. Louis
GARCH: Generalized Autoregressive Conditional Heteroskedasticity
GJRGARCH: The Glosten-Jagannathan-Runkle GARCH
IEMV: Infectious Disease Equity Market Volatility Index
KPSS: Kwiatkowski–Phillips–Schmidt–Shin
PP: Phillips-Perron
TGARCH: Threshold GARCH
VaR: Value at Risk
VIX: Volatility Index

## References

[1] Fernandes N. Economic effects of coronavirus outbreak (COVID-19) on the world economy. Available at SSRN 3557504. 2020.

[2] WongG, LiuW, LiuY, ZhouB, BiY, Gao GeorgeF. MERS, SARS, and Ebola: The Role of Super-Spreaders in Infectious Disease. Cell Host & Microbe. 2015;18(4):398–401.2646874410.1016/j.chom.2015.09.013PMC7128246

[3] BaldwinR, Di MauroBW. Economics in the Time of COVID-19. CEPR Press VoxEUorg eBook. 2020.

[4] Wilson A, Campos R, Shah I. Pandemics and the stock market. CSUS 30, April 2020, Sacramento USA. 2020.

[5] Hassan TA, Hollander S, van Lent L, Tahoun A. Firm-level exposure to epidemic diseases: Covid-19, SARS, and H1N1. National Bureau of Economic Research; 2020. Report No.: 0898–2937.

[6] ChenC-D, ChenC-C, TangW-W, HuangB-Y. The Positive and Negative Impacts of the Sars Outbreak: A Case of the Taiwan Industries. The Journal of Developing Areas. 2009;43(1):281–93.

[7] ChenM-H, JangS, KimWG. The impact of the SARS outbreak on Taiwanese hotel stock performance: An event-study approach. International Journal of Hospitality Management. 2007;26(1):200–12. doi: 10.1016/j.ijhm.2005.11.004 32287849PMC7116915

[8] IchevR, MarinčM. Stock prices and geographic proximity of information: Evidence from the Ebola outbreak. International Review of Financial Analysis. 2018;56:153–66.10.1016/j.irfa.2017.12.004PMC714893838620259

[9] Al-AwadhiAM, AlsaifiK, Al-AwadhiA, AlhammadiS. Death and contagious infectious diseases: Impact of the COVID-19 virus on stock market returns. Journal of Behavioral and Experimental Finance. 2020;27:100326. doi: 10.1016/j.jbef.2020.100326 32292707PMC7144859

[10] Onali E. Covid-19 and stock market volatility. Available at SSRN 3571453. 2020.

[11] Yilmazkuday H. Covid-19 effects on the s&p 500 index. Available at SSRN 3555433. 2020.

[12] LiuH, ManzoorA, WangC, ZhangL, ManzoorZ. The COVID-19 outbreak and affected countries stock markets response. International Journal of Environmental Research and Public Health. 2020;17(8):2800. doi: 10.3390/ijerph17082800 32325710PMC7215540

[13] SharifA, AlouiC, YarovayaL. COVID-19 pandemic, oil prices, stock market, geopolitical risk and policy uncertainty nexus in the US economy: Fresh evidence from the wavelet-based approach. International Review of Financial Analysis. 2020;70:101496.10.1016/j.irfa.2020.101496PMC722752438620230

[14] HeQ, LiuJ, WangS, YuJ. The impact of COVID-19 on stock markets. Economic and Political Studies. 2020:1–14.

[15] GoodellJW, HuynhTLD. Did Congress trade ahead? Considering the reaction of US industries to COVID-19. Finance Research Letters. 2020:101578. doi: 10.1016/j.frl.2020.101578 32837361PMC7261360

[16] ConlonT, CorbetS, McGeeRJ. Are Cryptocurrencies a Safe Haven for Equity Markets? An International Perspective from the COVID-19 Pandemic. Research in International Business and Finance. 2020:101248. doi: 10.1016/j.ribaf.2020.101248 34170988PMC7271856

[17] ConlonT, McGeeR. Safe haven or risky hazard? Bitcoin during the Covid-19 bear market. Finance Research Letters. 2020;35:101607. doi: 10.1016/j.frl.2020.101607 32550843PMC7246008

[18] GoodellJW, GoutteS. Co-movement of COVID-19 and Bitcoin: Evidence from wavelet coherence analysis. Finance Research Letters. 2020:101625.10.1016/j.frl.2020.101625PMC976119036569647

[19] GoodellJ, GoutteS. Diversifying with cryptocurrencies during COVID-19. 2020.

[20] SunY, WuM, ZengX, PengZ. The impact of COVID-19 on the Chinese stock market: Sentimental or substantial? Finance Research Letters. 2021;38:101838.10.1016/j.frl.2020.101838PMC976118836569651

[21] XuL. Stock Return and the COVID-19 pandemic: Evidence from Canada and the US. Finance Research Letters. 2021;38:101872.10.1016/j.frl.2020.101872PMC976118936569655

[22] OkorieDI, LinB. Stock markets and the COVID-19 fractal contagion effects. Finance Research Letters. 2021;38:101640. doi: 10.1016/j.frl.2020.101640 32837366PMC7275187

[23] ChangC-P, FengG-F, ZhengM. Government Fighting Pandemic, Stock Market Return, and COVID-19 Virus Outbreak. Emerging Markets Finance and Trade. 2021:1–18.

[24] RahmanML, AminA, Al MamunMA. The COVID-19 outbreak and stock market reactions: Evidence from Australia. Finance Research Letters. 2021;38:101832.10.1016/j.frl.2020.101832PMC976119536569654

[25] AnhDLT, GanC. The impact of the COVID-19 lockdown on stock market performance: evidence from Vietnam. Journal of Economic Studies. 2021;48(4):836–51.

[26] ContessiS, De PaceP. The international spread of COVID-19 stock market collapses. Finance Research Letters. 2021:101894. doi: 10.1016/j.frl.2020.101894 34566529PMC8450777

[27] MazurM, DangM, VegaM. COVID-19 and the march 2020 stock market crash. Evidence from S&P1500. Finance Research Letters. 2021;38:101690. doi: 10.1016/j.frl.2020.101690 32837377PMC7343658

[28] Aloui D, Goutte S, Guesmi K, Hchaichi R. COVID 19’s impact on crude oil and natural gas S&P GS Indexes. Available at SSRN 3587740. 2020.

[29] Yan B, Stuart L, Tu A, Zhang T. Analysis of the Effect of COVID-19 on the Stock Market and Investing Strategies. Available at SSRN 3563380. 2020.

[30] AnyaK. Measuring COVID-19 Effects on World and National Stock Market Returns. The Journal of Asian Finance, Economics and Business. 2021;8(2):1–13.

[31] GlostenLR, JagannathanR, RunkleDE. On the relation between the expected value and the volatility of the nominal excess return on stocks. The journal of finance. 1993;48(5):1779–801.

[32] JoeH. Dependence modeling with copulas: CRC press; 2014.

[33] Sklar A. Fonctions de reprtition an dimensions et leursmarges. 1959.

[34] Manner H. Estimation and model selection of copulas with an application to exchange rates: Citeseer; 2007.

[35] JoeH. Multivariate models and multivariate dependence concepts: CRC Press; 1997.

[36] TawnJA. Bivariate extreme value theory: models and estimation. Biometrika. 1988;75(3):397–415.

[37] GenestC, Carabarín-AguirreA, HarveyF. Copula parameter estimation using Blomqvist’s beta. Journal de la Société Française de Statistique. 2013;154(1):5–24.

[38] HofertM, KojadinovicI, MächlerM, YanJ. Elements of copula modeling with R: Springer; 2019.

[39] PattonAJ. Modelling asymmetric exchange rate dependence. International economic review. 2006;47(2):527–56.

[40] PattonA. Copula methods for forecasting multivariate time series. Handbook of economic forecasting. 2: Elsevier; 2013. p. 899–960.

[41] Baker SR, Bloom N, Davis SJ, Terry SJ. Covid-induced economic uncertainty. National Bureau of Economic Research. 2020;0898–2937.

[42] BentesSR, MenezesR. Entropy: A new measure of stock market volatility? Journal of Physics: Conference Series. 2012;394:012033.

[43] KimYS, RachevST, BianchiML, FabozziFJ. Financial market models with Lévy processes and time-varying volatility. Journal of Banking & Finance. 2008;32(7):1363–78.

[44] Trinidad SegoviaJE, Fernández-MartínezM, Sánchez-GraneroMA. A novel approach to detect volatility clusters in financial time series. Physica A: Statistical Mechanics and its Applications. 2019;535:122452.

[45] HeX-Z, LiK, WangC. Volatility clustering: A nonlinear theoretical approach. Journal of Economic Behavior & Organization. 2016;130:274–97.

[46] TsaiI-C. Volatility clustering, leverage, size, or contagion effects: The fluctuations of Asian real estate investment trust returns. Journal of Asian Economics. 2013;27:18–32.

